The article "Serum Fetuin-A Levels in Patients with Cardiovascular Disease: A Meta-Analysis" was retracted in 2020. Reasons: unreliable results or conclusions; bias or lack of balance; concerns about a third party's involvement.

# Serum Fetuin-A Levels in Patients with Cardiovascular Disease: A Meta-Analysis

**DOI:** 10.1155/2014/691540

**Published:** 2014-10-16

**Authors:** Ze-Lin Sun, Qi-Ying Xie, Gong-Liang Guo, Ke Ma, Yuan-Yuan Huang

**Affiliations:** ^1^Department of Cardiology, Xiangya Hospital, Central South University, No. 87 Xiangya Road, Kaifu District, Changsha 410008, China; ^2^Department of Cardiovascular Medicine, China-Japan Union Hospital of Jilin University, Jilin 132000, China; ^3^Department of Pediatrics, the First Affiliated Hospital of Jilin University, Jilin 132000, China

## Abstract

*Background*. Fetuin-A (FA) suppresses arterial calcification, promotes insulin resistance, and appears to be elevated in patients with cardiovascular diseases (CVD), but the data is still inconsistent. To clarify the correlation between serum FA levels and the presence and severity of CVDs, we performed this meta-analysis. *Method*. Potential relevant studies were identified covering the following databases: PubMed, Embase, Web of Science, Cochrane Library, CISCOM, CINAHL, Google Scholar, China BioMedicine (CBM), and China National Knowledge Infrastructure (CNKI) databases. Data from eligible studies were extracted and included in the meta-analysis using a random-effects model. *Results*. Ten case-control studies, including 1,281 patients with CVDs and 2,663 healthy controls, were included. The results showed significant differences in serum levels of FA between the CVDs patients and the healthy controls (SMD = 1.36, 95%CI: 0.37–2.36, *P* = 0.007). Ethnicity-subgroup analysis implied that low serum FA levels are related to CVDs in Caucasians (SMD = 1.73, 95%CI: 0.20–3.26, *P* = 0.026), but not in Asians (SMD = 1.04, 95%CI: −0.33–2.40, *P* = 0.138). *Conclusion*. The data indicated that decreased serum FA level is correlated with the development of CVDs. FA might be clinically valuable for reflecting the progression of CVDs.

## 1. Introduction 

Cardiovascular disease (CVD) refers to any disorder which disturbs the cardiovascular system, and so forth [1]. The World Health Organization (WHO) has revealed that CVD has become the leading cause of mortality worldwide; more individuals die from CVD than from any other disorders each year (http://www.who.int/mediacentre/factsheets/fs317/en/). CVD's estimated mortality rate is 17.1 million per year, representing 29 percent of the overall deaths worldwide, and its total mortality possibly exceeds one hundred million [1, 2]. Moreover, according to American Heart Association Statistics Committee and Stroke Statistics Subcommittee, though its death rate has fallen since the 1970s, CVD remains the leading cause of mortality in developed countries [3]. Being an age-specific disorder, there is abundance of evidence to suggest that there are multiple risk factors for CVD, including tobacco smoking, air pollution from the solid fuels, hyperlipidemia, diabetes, consumption of alcohol and sugar, obesity, and family history [4–6]. Additionally, varying serum levels of several proteins such as nitroproteins and the C-reactive protein have been reported to be related to CVD, and the fetuin-A (FA) protein has recently been the target of an increasing number of investigated cardiovascular disease [1, 7, 8].

FA, also known as alpha-2-Schmid Heremans glycoprotein (AHSG), is a phosphorylated glycoprotein and a member of the fetuin group of serum binding proteins, which are all comprised of three O-linked and two N-linked oligosaccharide chains [9–11]. FA is primarily synthesized by the hepatocytes and can also be produced in other human organs such as the kidneys and the tongue [11]. Serving as a mediating signal for antagonizing growth factor, FA inhibits the mineralization of the skeletal matrix [12]. FA can also bind with cationic ions like calcium^2+^, indicating that it is capable of inhibiting ectopic calcification [13, 14]. In addition, as the endogenous inhibitor of tyrosine kinase, FA may be related to the presence of insulin resistance in the target tissues [15]. Due to its multiple functions, elevated or decreased serum FA concentrations may be tightly linked to the progression of various diseases, atherosclerosis, for instance [16, 17]. For these reasons, we hypothesized that decreased serum FA concentrations may directly limit cardiac functions by effectively promoting cardiac fibrosis and calcification and thus influence CVD progression [18]. Prospective research has recognized that low serum FA levels are a valid predictor of CVD [19, 20]. In contrast, controversial opinions have supported the idea that reduced plasma concentrations of FA may increase CVD risk by inducing adipocyte-linked inflammatory cytokines [21, 22]. Because of the existence of contradictory theories on this subject, we conducted the following meta-analysis on downregulated serum FA levels and its contributory effects on CVD.

## 2. Materials and Methods

### 2.1. Data Sources and Keywords

To identify all pertinent papers that assessed the correlations between serum FA expression levels and CVDs, we comprehensively searched PubMed, Embase, Web of Science, Cochrane Library, CISCOM, CINAHL, Google Scholar, China BioMedicine (CBM), and China National Knowledge Infrastructure (CNKI) databases up to May 30st, 2014, utilizing selected common keywords regarding FA and CVDs. The keywords we selected for our initial literature search were “alpha-2-HS-Glycoprotein” or “AHSG protein, human” or “AHSG” or “fetuin-A” or “fetuin A” or “alpha-2 Heremans Schmid glycoprotein” or “alpha2-HS-glycoprotein” or “Alpha-2 Heremans Schmid Glycoprotein” for the exposure factors and “Coronary Artery Disease” or “CAD” or “MI” or “myocardial infarct” or “myocardiac infarction” or “myocardium infarction” or “cardiac infarction” or “myocardia infarction” or “infarction myocardium” or “myocardial infarcted” or “heart infarction” or “Myocardial Infarction” or “acute myocardial infarction” or “Coronary Heart Disease” or “CHD” or “AMI” for the outcome factors. No restriction was set on the language of the paper. We then scanned the bibliographies of relevant articles manually to identify additional potentially relevant papers.

### 2.2. Selection Criteria

We searched throughout for human-associated case-control studies assessing the association of FA serum levels with CVDs and reporting the adjusted standardized mean differences (SMDs) and 95% confidence intervals (CI). We only extracted data from studies that supplied the sample number and sufficient information about serum levels of FA, and we excluded articles with incomplete, unavailable, or inappropriate clinicopathologic data or those regarding CVDs not confirmed by histopathologic examinations. In addition, only studies with at least 20 subjects were used in this meta-analysis. However, when the extracted studies had subjects who overlapped more than 50% with two or more papers, we only included the one whose sample size was the largest. Furthermore, after careful reexamination, only the newest or most complete study was included when extracted studies were published by the same authors or groups.

### 2.3. Data Extraction

In order to reduce bias and enhance credibility, two investigators extracted information from the retrieved papers according to the selection criteria separately and arrived at a consensus on all the items through discussion and reexamination. The following relevant data was extracted from eligible studies prospectively in the final analyses: surname of first author, year of publication, source of publication, source of controls, study type, study design, sample size, age, sex, ethnicity and country of origin, type of cardiovascular disease, detection method of FA serum levels, and the serum levels of FA in cases and controls. Both authors approved the final determination about which of the studies to include.

### 2.4. Quality Assessment

To decide whether the study in question was of high quality, the two authors used a set of predefined criteria based on the Newcastle-Ottawa scale (NOS) criteria to assess the studies independently [28]. The NOS criteria are scored based on three aspects: (1) subject selection: 0 ~ 4; (2) comparability of subject: 0 ~ 2; and (3) clinical outcome: 0 ~ 3. Total NOS scores range from 0 (lowest) to 9 (highest). According to the NOS scores, the included studies were classified into two levels: low quality (0–6) and high quality (7–9), respectively. Discrepancies on NOS scores of the enrolled articles were resolved by consultation with an additional reviewer.

### 2.5. Statistical Analysis

To calculate the effect size for each study, the summary SMDs with 95% CI were used for control versus case category of FA serum levels with the *Z* test. In order to supply quantitative evidence of all selected studies and minimize the variance of the summary SMDs with 95% CI, we utilized a random-effects model (DerSimonian and Laird method) or a fixed-effects model (Mantel-Haenszel method) of individual study results when data from independent studies could not be combined. The random-effects model was applied when heterogeneity existed among studies, and the fixed-effects model was applied when there was no statistical heterogeneity. The subgroup meta-analyses were also conducted by ethnicity and sample size to explore potential effect modification. Heterogeneity amongst the enrolled studies was evaluated by Cochran's *Q*-statistic (*P* < 0.05 was regarded as statistically significant) [29]. Because of the low statistical power of the Cochran's *Q*-statistic, the *I* ^2^ test was also used to measure the possibility of heterogeneity between studies [30]. The *I* ^2^ test values ranged from 0% (no heterogeneity) to 100% (maximal heterogeneity). One-way sensitivity analysis was performed by deleting single studies included in our meta-analysis one by one to evaluate whether the results could have been significantly affected. A funnel plot was constructed to assess publication bias which might affect the validity of the estimates. The symmetry of the funnel plot was further evaluated by Egger's linear regression test [31]. All tests were two-sided and a *P* value of <0.05 was regarded as statistically significant. To make sure that the results are credible and accurate, two investigators input all information in the STATA software version 12.0 (Stata Corp, College Station, TX, USA) separately and arrived at an agreement.

## 3. Results

### 3.1. Included Studies

Our present meta-analysis included a total of 10 case-control papers published between 2002 and 2014 that evaluated the correlation of FA serum levels with CVDs in Asian (4 studies) and Caucasian populations (6 studies), including 1,281 patients with CVDs and 2,663 healthy controls, [10, 19–27]. The characteristics and methodological quality of the extracted studies are presented in Table 1. The countries where the studies were performed were Greece, China, Italy, Hungary, Turkey, Germany, France, and USA. Turkey was the country in which the largest number of studies was conducted (*n* = 3). The sources of controls in our present meta-analysis were mostly population-based (PB) studies and several hospital-based (HB) studies. The diseases considered in our meta-analysis were coronary artery disease (CAD), CAD with T2DM, acute coronary syndrome (ACS), ST-elevation myocardial infarction (STEMI), myocardial infarction (MI), stable angina (SA), and acute myocardial infarction (AMI). The methods for detecting FA serum levels in this meta-analysis included radioimmunoassay (RIA) and enzyme linked immunosorbent assay (ELISA). ELISA was used most frequently in the studies included in our meta-analysis. As for screening the studies, a flow chart of the study selection process is displayed in Figure 1. Initially, a total of 133 papers were selected from the 9 databases through based on the title and key words. After excluding the duplicates (*n* = 2), letters, reviews or meta-analysis (*n* = 15), non-human studies (*n* = 19), and the studies not related to research topics (*n* = 24), the remaining studies (*n* = 73) were reviewed and additional 58 studies were excluded because they were not case-control or cohort studies (*n* = 12), not relevant to FA (*n* = 21), or not relevant to CVDs (*n* = 25). After reviewing the remaining 15 trails, 10 papers were selected for the final analysis. During the final selection process, the major reason for rejection was that the studies did not supply enough information (*n* = 5). From 2001 to 2014, the number of articles selected from those electronic databases is shown in Figure 2.

### 3.2. Effect of FA Serum Levels on CVDs

As shown in Figure 3, our meta-analysis revealed a positive association between low FA serum level and CVDs (SMD = 1.36, 95% CI: 0.37–2.36, *P* = 0.007). Subgroup analysis based on ethnicity implied that low FA serum levels may be the main risk factor for CVDs in Caucasian populations (SMD = 1.73, 95% CI: 0.20–3.26, *P* = 0.026), but not in Asian populations (SMD = 1.04, 95% CI: −0.33–2.40, *P* = 0.138) (as shown in Figure 4). Further subgroup analyses by sample size showed that FA serum levels were positively correlated with CVDs in both large sample (SMD = 1.51, 95% CI: 0.26–2.76, *P* = 0.018) and small sample subgroups (SMD = 1.07, 95% CI: 0.51–1.62, *P* < 0.001) (as shown in Figure 4).

### 3.3. Sensitivity Analysis and Publication Bias

A leave-one-out sensitivity analysis was carried out to evaluate the stability of this meta-analysis. Each study included in our meta-analysis was evaluated one by one to reflect the effect of pooled SMDs. The overall statistical significance did not change when any single study was omitted. Therefore, the data presented in this meta-analysis is relatively stable and credible (Figure 5). The graphical funnel plots of the 10 included studies showed a slight asymmetry, and Egger's test showed publication bias (both *P* < 0.001) (Figure 6).

## 4. Discussion

Based on the results of our analysis, we claim that there is a significant connection between lower serum levels of FA and CVDs. With three O-linked and two N-linked chains of oligosaccharides, FA secreted in the liver, especially under the condition of hepatic steatosis, binds with bioactive Ca^2+^. This suggests that FA is a potential inhibitor of systemic calcification [10]. Additionally, FA could inhibit the inflammatory response self-amplification by improving the uptake of cationic inhibitors in the synthesis of proinflammatory cytokine [22]. Furthermore, FA could also prevent the autophosphorylation of insulin receptors and the activity of tyrosine kinase (an insulin receptor), which might be a risk for the development of type 2 diabetes [26]. However, it should be noted that with respect to the role of preventing insulin resistance, it cannot be regarded as the direct factor related to the development of CVDs, since insulin resistance is significantly correlated with the production of insulin and then the abnormality of lipid, whereas the predominant reason for CVDs is atherosclerosis [32]. Aside from its role in preventing insulin resistance, FA also has a relationship with metabolic syndrome, atherogenic dyslipidemia and reduced adiponectin levels, and risk factors for nonalcoholic fatty liver disease and might also be involved in fibrosis of liver [21]. Based on this information, there is an apparent contradiction in the fact that low levels of fetuin-A are associated with CVD while high levels are associated with NAFLD and diabetes [29, 33]. Many studies have shown that lower serum levels of FA have a close connection with CVDs, such as CAD, MI, ACS, and S-T STEMI [18, 25]. The function of FA as an inhibitor of calcification and connection with arterial stiffness, intimal-medial thickness, and changes in the arterial wall indicates that FA does have a role in calcified coronary artery disease. Moreover, Mori et al. have shown that lower serum levels of FA are correlated with the disease [34]. Lower serum levels of FA could promote inflammatory processes and the production of cardiotoxic TNF, resulting in left ventricle remodeling and acute coronary syndrome relapse [24]. Based on the above facts, we can conclude that lower serum levels of FA play an important role in the development of CVDs because of the function of FA in systemic calcification and inflammatory process. In agreement with our study, Kanbay et al. have found abnormal serum levels of FA in the early course of CAD in a young group with mild-to-moderate kidney function alteration, suggesting that there is an independent biomarker for CAD development [35]. However, there were also some studies demonstrating the relationship of high level of FA and the development of CVD [26, 36]. The possible mechanisms lied in the fact that FA could promote atherosclerosis in CVD patients through insulin resistance induction and promote the expression of cytokine in monocytes to participate in the inflammation [10]. The contradiction conclusion in the studies might be due to the influence of diabetes on the relationship of FA serum level and the development of CVD, because some subjects are CVD patients with diabetes; the higher level of FA might mainly be due to the diabetes. Thus the accuracy of the contradictory conclusion is susceptible.

Given the fact that some other related factors may participate in the connection between lower serum levels of FA and CVD patients, a stratified analysis based on ethnicity and sample size was conducted. From the stratified analysis based on ethnicity, we discovered that the relationship is significant among Caucasians but not Asians. This might be explained by different living backgrounds and different genetic factors between the two races. In summary, our results are partly inconsistent with other studies which have shown that the serum level of FA is inversely associated with the development of CVDs, suggesting that FA is significant and useful marker for the development and progression of CVDs.

Our study had several limitations. Firstly, we included four studies that have a limited number of patients which might have impaired the statistical power of analysis, and therefore, results of our meta-analysis need to be confirmed by studies with larger sample sizes. Secondly, we cannot rule out the impacts of individuals' body mass index (like the difference in blood pressure and cholesterol) and lifestyle differences on the results. Third, only serum FA levels were examined in the current meta-analysis which may be insufficient to confirm our viewpoints; hence, additional research on other inflammatory biomarkers in the same samples could provide more valuable information on this association. Finally, considering that this is a typical cross-sectional epidemiological study and not a prospective investigation on this relationship, no final conclusion with respect to causality and temporality of the explored connection can be drawn. Thus, the information we used was insufficient for precluding the possibility of an inconsistent outcome in the future.

In summary, serum FA levels were possibly related to the presence and severity of CVDs. Our current cross-sectional analysis may not address certain key issues comprehensively. Hence, prospective cohort studies will be conducted to answer the question of the influence of serum FA levels on CVDs.

## Figures and Tables

**Figure 1:** Flow chart shows study selection procedure. Thirteen case-control studies were included in this meta-analysis.

**Figure 2:** The distribution of the amount of articles in electronic databases over the last decade.

**Figure 3:** Forest plots on the difference of serum fetuin-A levels between cardiovascular disease patients and healthy subjects.

**Figure 4:** Subgroup analyses on the difference of serum fetuin-A levels between cardiovascular disease patients and healthy subjects.

**Figure 5:** Sensitivity analysis of the summary odds ratio coefficients on the difference of serum fetuin-A levels between cardiovascular disease patients and healthy subjects.

**Figure 6:** Funnel plot of publication biases on the difference of serum fetuin-A levels between cardiovascular disease patients and healthy subjects.

**Table 1:** Characteristics of included studies focused on serum levels of FA.

First author	Year	Ethnicity	Sample size		Gender (M/F)		Age (years)		Disease	Method	Main finding	Mean value (ug/mL)	NOS score
			Case	Control	Case	Control	Case	Control				(Case versus control)	
Kadoglou [20]	2014	Caucasians	95	35	68/27	28/7	67.1 ± 6.5	65.0 ± 9.5	CAD	ELISA	①	222.00 versus 839	7
Zhao [10]	2013	Asians	129	69	67/62	35/34	63.1 ± 8.9	62.9 ± 9.0	CAD with T2DM	ELISA	②	451.14 versus 396.41	7
			129	69	67/62	35/34	63.1 ± 8.9	62.9 ± 9.0	CAD with T2DM	ELISA		451.14 versus 308.3	
Ballestri [21]	2013	Caucasians	46	24	35/11	13/11	67.6 ± 11.4	68.9 ± 13.6	CAD	ELISA	③	374 versus 445.8	6
Voros [23]	2012	Caucasians	171	81	120/51	46/35	62.0 ± 6.0	60.0 ± 7.0	MI	RIA	④	673 versus 673	8
Afsar [24]	2012	Asians	95	81	68/27	32/49	61.8 ± 12.1	48.3 ± 9.2	ACS	ELISA	⑤	760 versus 1100	7
Basar [19]	2011	Asians	180	55	152/28	46/9	57.9 ± 9.4	56.7 ± 8.2	STEMI	ELISA	⑥	286.85 versus 359.8	8
Bilgir [25]	2010	Asians	34	42	—	—	60.3 ± 11.8	59.6 ± 11.9	MI	ELISA	⑦	156 versus 179	5
							59.4 ± 8.8	59.6 ± 11.9	SA	ELISA		167 versus 179	
Weikert [26]	2008	Caucasians	227	2198	164/63	798/1400	57.5 ± 0.6	49.5 ± 0.2	MI	ELISA	⑧	253.6 versus 226.9	8
Lim [22]	2007	Caucasians	284	34	233/51	20/14	60.0 ± 14.0	67.0 ± 14.0	STEMI	ELISA	⑨	188 versus 219	8
Mathews [27]	2002	Caucasians	20	44	14/6	23/21	55 (43~69)	48 (38~62)	AMI	ELISA	⑩	281.3 versus 312.3	6

FA: fetuin-A; M: male; F: female; CAD: coronary artery disease; MI: myocardial infarction; ACS: acute coronary syndrome; STEMI: ST-elevation myocardial infarction; SA: stable angina; AMI: acute myocardial infarction; NOS: Newcastle-Ottawa Scale; ①: derangements in serum levels of all vascular calcification inhibitors compared with those in healthy controls. Simvastatin treatment for 6 months significantly decreased serum fetuin-A, OPG, and OPN levels; ②: serum fetuin-A levels are independently correlated with the presence and severity of CAD in T2DM patients; ③: high fetuin-A levels are independently associated with NAFLD and a lower risk of chronographically diagnosed CAD; ④: ghrelin level is determined by elevated insulin and decreased adiponectin levels; ⑤: fetuin-A levels decrease in patients with acute coronary syndromes, independent of heart valve calcification; ⑥: low-admission fetuin-A levels are associated with impaired coronary flow in STEMI patients undergoing primary percutaneous coronary intervention; ⑦: fetuin-A levels seem to be decreased in SA and MI patients; ⑧: high plasma fetuin-A levels are correlated with an increased risk of MI and IS; ⑨: fetuin-A is an important predictor of death at 6 months in STEMI patients independent of NT-proBNP, CRP, and CADILLAC risk score; ⑩: Plasmaa2-HSG concentrations start to decrease within a few hours after the onset of AMI and return to near normal concentrations during the recovery period (5–7 days after AMI).
